RETRACTED

# Sentiment Analysis on COVID-19 Twitter Data Streams Using Deep Belief Neural Networks

**DOI:** 10.1155/2022/8898100

**Published:** 2022-05-06

**Authors:** Jatla Srikanth, Avula Damodaram, Yuvaraja Teekaraman, Ramya Kuppusamy, Amruth Ramesh Thelkar

**Affiliations:** ^1^Department of Computer Science and Engineering, Aurora's Technological and Research Institute, Hyderabad 500098, TS, India; ^2^School of Information Technology (SIT), JNTUH, Hyderabad 500085, TS, India; ^3^Department of Electronic and Electrical Engineering, The University of Sheffield, Sheffield S1 3JD, UK; ^4^Department of Electrical and Electronics Engineering, Sri Sairam College of Engineering, Bangalore 562106, India; ^5^Faculty of Electrical & Computer Engineering, Jimma Institute of Technology, Jimma University, Jimma, Ethiopia

## Abstract

Social media is Internet-based by design, allowing people to share content quickly via electronic means. People can openly express their thoughts on social media sites such as Twitter, which can then be shared with other people. During the recent COVID-19 outbreak, public opinion analytics provided useful information for determining the best public health response. At the same time, the dissemination of misinformation, aided by social media and other digital platforms, has proven to be a greater threat to global public health than the virus itself, as the COVID-19 pandemic has shown. The public's feelings on social distancing can be discovered by analysing articulated messages from Twitter. The automated method of recognizing and classifying subjective information in text data is known as sentiment analysis. In this research work, we have proposed to use a combination of preprocessing approaches such as tokenization, filtering, stemming, and building *N*-gram models. Deep belief neural network (DBN) with pseudo labelling is used to classify the tweets. Top layers of the base classifiers are boosted in the pseudo labelling strategy, whereas lower levels of the base classifiers share weights for feature extraction. By introducing the pseudo boost mechanism, our suggested technique preserves the same time complexity as a DBN while achieving fast convergence to optimality. The pseudo labelling improves the performance of the classification. It extracts the keywords from the tweets with high precision. The results reveal that using the DBN classifier in conjunction with the bigram in the *N*-gram model outperformed other models by 90.3 percent. The proposed approach can also aid medical professionals and decision-makers in determining the best course of action for each location based on their views regarding the pandemic.

## 1. Introduction

The new coronavirus illness (COVID-19) is an ongoing pandemic that has sparked widespread concern around the world. Spreading misleading information on social media platforms like Twitter, on the other hand, is exacerbating the disease's concern. People can stay safe, informed, and connected with the help of technological improvements and social media. The same instruments, on the other hand, enable and intensify the current infodemic, which continues to undermine the global response and risk pandemic-control measures. Despite the fact that young people are at a lower risk of serious sickness from COVID-19, they are an important group in the context of the pandemic and share in the communal responsibility of helping us stop transmission. They are also the most active online, using different digital channels per day (such as Twitter, Facebook, TikTok, WeChat, and Instagram).

RETRACTED

Social media has swiftly grown into a crucial communication tool for the production, transmission, and consumption of information since the start of the COVID-19 epidemic. Several studies have already used social media data to aid in the detection and identification of infectious disease epidemics, as well as the interpretation of public attitudes, behaviours, and perceptions. As social media content is provided by users, it can be subjective or erroneous, and it commonly contains misinformation and conspiracy theories [1]. Sentiment analysis, also known as opinion mining, is the method of classifying emotions in subjective data using machine learning (ML) and natural language processing (NLP).

By analysing and sharing information from peer-reviewed, published research, policymakers and public health organizations may design efforts for accurate and timely knowledge translation to the general population. Individual profiles have evolved, reinforced by social networks, which have had a similar influence on the more specialized communication medium, in addition to traditional media as the main drivers of social communication in crisis situations. The findings suggest to set a new communications paradigm that creates a new area for agents whose material has a level of engagement equivalent to, if not greater than, that of digital health media [2].

The current COVID-19 problem is resulting in a socially advanced condition that is unprecedented for health communities. We live in a highly globalized society, where mobility, unrestricted travel between countries, and the evolution and application of Information and Communication Technologies (ICTs) are all highly developed. Similarly, there is a continual stream of bogus news and criticism of movements on social media sites as a result of the viral pandemic. It stifles public health professionals' communication and incites broad public indignation [3].

RETRACTED

A convolutional neural network (CNN or ConvNet) is a type of deep neural network used to interpret visual imagery in deep learning. Artificial neural networks have ushered in new ideas and procedures in machine learning in a variety of fields during the last two decades. Many existing processes have been replaced by them. ConvNets are made up of filter layers (known as convolutional layers) and aggregation layers (known as pooling layers), which are alternately repeated. One or more fully connected layers follow them.

Text classification aims to categorize text documents into one or more predetermined categories automatically. Understanding audience sentiment (happy, sad, and furious) from social media, detecting spam and nonspam emails, auto tagging of customer enquiries, categorization of news items into predetermined subjects, and so on are some instances of text classification [4].

Text encoders are generally pretrained to handle text as a sequence of tokens corresponding to small text units, such as English word parts. In many NLP jobs, where a powerful encoder is required to model more contextual information, a high quality of text representation plays a key part in achieving good performance. Text mining and information retrieval need the selection of text feature items, which is a fundamental and significant task. Deep learning differs from traditional methods in that it automatically learns features from huge data rather than adopting handmade characteristics, which rely heavily on past knowledge of designers and make it nearly impossible to take advantage of massive data [5]. Text classification framework using a supervised learning model is shown in Figure 1.

The deep counterpart of an auto encoder is a stacked auto encoder, which may be produced simply by stacking layers. The learnt representation of the previous layer is the input for each layer, and it learns a more compact representation of the existing learned representation. We propose to use feature extraction from the twitter data streams using *n*-gram stack encoder followed by setting the rules and training the neural network for classifying streaming data. We will concentrate on the data stream classification task, where the parameters of a classification model may change over time, requiring the model to adapt.

## 2. Related Work

The COVID-19 pandemic has resulted in a massive loss of human life around the world and poses a significant threat to global health, food chain, and the workplace. The COVID-19 epidemic has claimed many lives and poses a serious danger to world health, the food supply, and the workplace. The response differences between social media and financial markets as a result of the severe viral spread's after-effects revealed the dynamics of COVID-19, including mortality, contagion variables, time of country virus, and early fatalities. During the lockdown, social media channels were critical in spreading information about the pandemic around the world, as people used the platforms to express their emotions. In light of this severe situation, it is necessary to examine people's reactions on Twitter, taking into consideration popular words that are directly or indirectly related to the epidemic [6].

RETRACTED

It would be practically impossible for a human to read and comprehend everything that has been said about COVID-19 vaccinations on Twitter. Fortunately, using textual feature extraction, sentiment analysis, and word cloud visualizations, we can look into an incredibly complicated and wide-ranging dialogue using natural language processing (NLP) approaches. Bhatia et al. made a study on sentiment analysis of COVID-19 tweets with the help of deep learning classifiers [7]. People were not guided by tweets about the COVID-19 epidemic, according to this research. The findings show that neither WordCloud nor the frequency of terms in tweets contains any useful words. A proposed deep learning classifier model with an accuracy of up to 81 percent validates the claims. The authors claim that a fuzzy rule based on Gaussian membership correctly recognizes sentiments from tweets.

Amit et al. have proposed a sentiment analysis on the impact of coronavirus in social life using the BERT model. They claim that, because Twitter has become one of the most prominent social media sites, the authors conducted sentiment analysis on tweets using the BERT model, based on people's excitement and opinions to better understand their mental state [8]. The authors conducted a sentiment analysis on two data sets in this paper: one data set contains tweets from people all over the world, while the other data set contains tweets from people in India. They used the GitHub repository to validate the emotion classification's accuracy. The validation accuracy is 94 percent, according to the experimental data.

With the growth in COVID-19 cases, a strange position of pressure was placed on each country to manage the problem and make the best use of available resources. People experienced panic, anxiety, and depression as the number of positive cases increased rapidly around the world. The impact of this lethal disease was discovered to be directly proportionate to the population's physical and mental health. Social media has been the most prominent tool that has disrupted human life during this period. The tweets about COVID-19, whether they were about a large number of positive cases or deaths, caused a surge of panic and concern among people all across the world. Researchers and data scientists will be able to access the data for academic and research purposes. Many data points related to real-life occurrences, such as COVID-19, can be found in social media data. Harleen Kaur and others have used the R programming language to analyse the Twitter data. The authors gathered data from Twitter using hashtag terms such as COVID-19, coronavirus, deaths, new case, and recovered cases. They used an algorithm called hybrid heterogeneous support vector machine (H-SVM) for sentiment classification and categorised the scores as positive, negative, or neutral in this study [9]. They also compared the suggested algorithm's performance to that of the recurrent neural network (RNN) and support vector machine on specific criteria such as precision, recall, *F*1 score, and accuracy (SVM).

RETRACTED

In a very short period of time, the social networking site Twitter saw an extraordinary rise in tweets pertaining to the novel Coronavirus. Gurumurthy et al. conducted a global sentiment analysis of coronavirus tweets, demonstrating how public opinion in various nations has changed over time. Furthermore, tweets relating to work from home (WFH) and online learning were scraped and the change in sentiment over time was studied to identify the impact of coronavirus on daily elements of life. The authors also tested the accuracy of several machine learning models for sentiment categorization, such as long short term memory and artificial neural networks [10].

Kuhn et al. have discussed cross-language sentiment analysis of European Twitter messages during the COVID-19 pandemic in their work. The difficulty in analysing the data source stems from the fact that social media communications are exceedingly noisy and idiosyncratic, and the volume of incoming data is far too enormous to manually evaluate. As a result, the authors found that automated methods for extracting useful information are required. The authors examine the emotion of Twitter messages collected during the first months of the COVID-19 outbreak in Europe [11]. This is done utilizing multilingual sentence embedding and a neural network for sentiment analysis. The researchers categorize the findings by place of origin and compare their chronological progression to events in those countries. This allows them to investigate how the situation affects people's moods. They discovered, for example, that lockdown announcements are associated with a drop in mood in almost all of the countries studied, which recovers quickly.

RETRACTED

Anupam Mondal and others have presented a new approach to classify COVID-19 tweets using machine learning algorithms. The documentation goes over the methods for preprocessing tweets, feature extraction, and developing machine learning models in detail. When the organizers evaluated both of the created learning models, they received *F*1 ratings of 0.93 and 0.92, respectively [12]. They passed the words, POS tags, and TF-IDF values through their default TensorFlow embedding layer as separate inputs, then concatenated the outputs to train the DL model. The output of the concatenation layer was then sent to a dense layer that mapped the tensors to their labels via two layers of bidirectional long-short term memory.

Ching have proposed a *n*-Gram statistics for natural language understanding and text processing [13]. For applications in natural language understanding and text processing, *n*-gram statistics and other features of the English language were determined. They were calculated using 1 million word samples from a well-known corpus. Similar features were discovered in three more corpuses' most frequently used 1000 words. The *n*-gram positional distributions produced in this investigation are discussed. There are statistical studies on word length and *n*-gram frequency trends versus vocabulary. A collection of *n*-gram statistics obtained by different researchers is evaluated and compared in addition to a study of *n*-gram statistics found in the literature.

With the recent growth of data in motion, there is a rising academic interest in analysing streaming data, which has resulted in the publication of numerous new papers on data stream analytics. But, investigating the capabilities of traditional recurrent neural networks in the context of streaming data classification is still a relatively unexplored area. Monidipa Das et al. have presented a model called FERNN, a unique RNN variant with single-pass learning capability and self-evolution attribute [14]. FERNN is well suited to working with streaming data due to its online learning abilities, while its self-organizing trait makes it adaptable to a fast changing environment. In the hidden layer, FERNN employs hyperplane activation, which not only reduces network parameters but also causes the model to act as a teacher forcing mechanism by default, automatically addressing the vanishing/exploding gradient issues that can arise with traditional RNN learning based on back-propagation-through-time policy. As it is not limited by the normal distribution assumption for streaming data, FERNN is more flexible than the majority of the existing autonomous learning models. Under the test-then-train approach, the efficacy of FERNN is assessed in terms of classifying six publicly available data streams. The experimental findings suggest that FERNN can achieve state-of-the-art classification accuracy with a relatively low computation cost.

RETRACTED

A methodology is proposed to analyse COVID-19 from Arabic twitter tweets. Naïve Bayes classification is used for basic classification. Later ensemble methods are used for analysis. Ensemble methods with SMOTE is performed better than basic classifiers [15]. The polarization is performed using machine learning algorithms, deep learning, and TextBlob. The deep learning approach such as Bi-LSTM performed when compared to other methods [16]. People emotions are analysed and classified as positive, negative, and neural. The machine learning algorithms, deep learning algorithms, and ensemble methods are used [17].

In this work, we propose to use a feature extraction using *n*-gram stack encoder method first. Data collection and preprocessing are the first steps in our research work. The preprocessing involves different phases including data cleaning, finding polarity, finding sentiments, and combining the data sets. To get the sentiments, we then use different methods including parts of speech tagging, lemmatization, stemming, stop words removal, and finding the keywords. Once the features are extracted, we then use the convolutional neural network for classifying the streaming data. In machine learning, we utilize the deep belief neural network, which is a generative graphical model, or a form of deep neural network, made up of several layers of latent variables with connections between levels but not between units within each layer. Our results are found to be promising and better as compared to the existing methods in the literature that we have discussed in this section.

## 3. Data Collection and Preprocessing

Businesses may interact with customers on Twitter in a more personal way. However, because Twitter has so much data, it can be difficult for marketers to pick which tweets to respond to first. As a result, sentiment analysis has become an important tool in social media marketing campaigns. Sentiment analysis is a technique that automatically tracks sentiments in social media interactions. Data collection is the first step in this research problem of sentimental analysis of the COVID-19 twitter data [18]. To follow certain terms and accounts that were trending at the time of data collection, we used Twitter's streaming application programming interface (API) and Tweepy. There are several steps involved in the process of using Twitter's API to build the data set. This includes creating an account, installation of Tweepy, a quick test run, inspecting a tweets JSON, parsing out the data, identifying and collecting the data. Once the data are collected, it should be preprocessed before further steps.

RETRACTED

Both data preprocessing and exploratory data analysis are included in the second phase. The raw tweets were incapable of creating unbiased results in sentiment prediction during the process of cleaning the data to uncover useable characteristics. #tags, @mentions, URLs, and stop words in tweets were the biggest roadblocks. Regular expression-based substitution were used to remove the #tags, @mentions, and URLs from the tweets. Stop words were handled by NLTK library in python.

The polarity scores of each tweet in the dataset can be computed using Python's TextBlob package [19]. The cleaned tweets from the previous phase were subjected to multiple assessment models using TextBlob, and a generic polarity score for each tweet was calculated. This score was linked to the type of words in the text, such as Unigrams, Bigrams, and Trigrams.

By classifying the polarity ratings of tweets into three groups, the sentiments phase expanded on the preceding phase. Positive emotions are ones that have a wide range (0, 1). Negative sentiments have a polarity of (−1, 0), while neutral sentiments have a polarity of 0.0. These three classes were saved in the dataset as a separate feature called “Sentiments.” Parts of speech tagging (POS), lemmatization, stemming, and stop words removal were the different techniques used in the framework process as shown in Figure 2.

A part-of-speech tag (or POS tag) is a particular label assigned to each token (word) in a text corpus to denote the part of speech as well as other grammatical categories such as tense, number (plural/singular), and case [20]. POS tags are employed in text analysis tools and algorithms, as well as in corpus searches.

In linguistics, lemmatization is the act of bringing together the inflected forms of a word so that they may be examined as a single item, identified by the word's lemma, or dictionary form [21]. The process of reducing inflected words to their word stem, base, or root form, generally a written word form, is known as stemming. The stem does not have to be the same as the word's morphological root; it is typically enough that related words map to the same stem, even if that stem is not a valid root in and of itself. To eliminate stop words from a sentence [22], divide your text into words and then check to see if the word is in the NLTK list of stop words.

All things in Twitter are built on the foundation of tweets. “Status updates” is another term for tweets. The Tweet object has a huge list of “root-level” characteristics, including id, created at, and text, among others. Tweet objects also serve as the “parent” object for a number of child objects. The key attributes from the tweets include the following:

- text: the tweet's actual text
- created at: the date the tweet was created
- text: the text of the tweet itself
- favorite count, retweet count: the total number of favourites and retweets favorited
- lang: the language's abbreviation
- id: the tweet identifier
- geo: if available, geo-location data
- user: author's complete profile
- entities: URLs, @-mentions, hashtags, and symbols are examples of entities

Data preparation is highly recommended for a variety of reasons, including datum or database quality, data analysis process, and the capacity to apply related algorithms for removing noisy and missing data and increasing data reliability, as high-quality data models require high-quality data. Sentiment analysis entailed determining the subjectivity contents of a given piece of material by first preprocessing it to detect stop words and symbols and then checking the subjectivity contents [23]. Machine learning approaches and lexical-based methods are both used to determine the polarity of an opinion's substance. Sentiment classifies information as either favourable, negative, or neutral.

RETRACTED

Feature selection is a method for condensing a large number of attributes into a smaller subset with the maximum accuracy [24]. The limitation of overfitting, the improvement of accuracy, and the reduction in training time are all advantages of using this option on the data. Filters and wrappers are two types of feature selection strategies. Filters utilize statistical tests like Infogain, Chi-square, and CFS to determine the best subset of features, whereas wrappers use a learning algorithm to determine the best subset of features.

In the literature, the majority of comprehensive techniques extract unigrams, bigrams, and unigrams and bigrams as three separate features to apply to Naive Bayes, maximum entropy, and support vector machines classifiers, respectively [25]. *N*-grams features have been frequently employed in twitter sentiment classification to speed up processing speed. In more concrete terms, information gain for classification is a measure of how frequently a feature appears in one class compared to all other classes. A unigram with high information is one that appears frequently in good tweets and rarely in negative tweets. In the next section, we detail the proposed approach through *n*-gram stack encoder followed by setting the rules and training the neural network for classifying streaming data.

RETRACTED

## 4. Proposed Design

Sentiment analysis is an automated approach of identifying and classifying subjective information in text data. An opinion, a judgment, or a visceral response to a particular issue or element of a product might be included. Polarity detection is the most popular method of sentiment analysis, which involves categorizing statements as positive, negative, or neutral. Sentiment analysis makes sense of human language using natural language processing and machine learning to produce correct results automatically. Connect sentiment analysis tools directly to social networks so that we can keep track of tweets as they come in and obtain real-time insights from social mentions.

We focus on an automatic method for sentiment analysis in order to examine these vast amounts of data. For sentiment analysis on tweets, we train a neural network. A pretrained word embedding follows the network's text input layer. The vectors are then input into a 128-dimensional fully connected layer with 50% dropout and sigmoid activation, followed by a regression output layer.

An *n*-gram is an *n*-unit string that is a portion of a bigger string. Characters and entire words can be used as these units. A word is just a string of *x* characters separated by a space on both sides. Because word borders are also essential information, spaces are usually included when utilizing character *n*-grams for classification.

An *n*-gram is a contiguous sequence of *n* elements from a given sample of text or speech in the fields of computational linguistics and probability as shown in Figure 3. The components might be phonemes, syllables, letters, words, or base pairs, depending on the application. *n*-grams are often retrieved from a text or audio corpus. *N*-grams are also known as shingles when the components are words. In statistical natural language processing, *n*-gram models are commonly utilized. Words are modelled in such a way that each *n*-gram is made up of *n* words for parsing.

The lack of explicit representation of long-range dependency in *n*-gram models is frequently criticized [26]. Because an *n*-gram model's only stated dependency range is (*n* − 1) characters and because natural languages contain many occurrences of unbounded dependencies, an *n*-gram model cannot discriminate unbounded dependencies from noise in principle. But in practice, *n*-gram models have proven to be particularly effective in modelling language data, which is a critical component of modern statistical language applications.

In general, word-level *N*-grams give “better” outcomes for generative applications, but they come with their own set of problems. An *N*-Gram grammar is a representation of a *N*th order Markov language model in which the existence of *N* − 1 extra symbols affects the chance of a symbol appearing. Word sequence probabilities are derived by the cooccurrences of words in the corpus, and *N*-Gram grammars are frequently created using data taken from a huge corpus of text. *N*-Gram grammars have the advantage of covering a considerably bigger language than would customarily be possible with a corpus-based approach.

RETRACTED

When you count the number of *n*-grams shared by two strings, you get a measure of how similar they are. This metric is impervious to a wide range of textual errors, including misspellings. *n*-grams are commonly used as features in machine learning to predict the particular qualities of components in a dataset.

All of the tweets in the training set can be transformed to *n*-grams in the case of hashtag prediction. After that, *n*-gram frequency counts, for example, might be used to find patterns in the data. Specific hashtags could be linked to specific *n*-gram frequencies for tweets. A hashtag prediction system of maximum possibilities can be created in this fashion. A method like this might also extract all *n*-grams inside a specific range.

The amount of unique words identified in the training data determines the number of features in normal circumstances. The program can extract *n*-grams at both the character and word level. Other settings in this method can be predetermined, such as omitting stop words and non-ASCII letters. The non-ASCII letter should be removed before sentiment analysis to improve the performance.

### 4.1. Algorithm

We will begin with the uniform model. Because it assigns the same probability to every word in the text, this model will have very low average log likelihoods on the evaluation texts. After that, we combine this uniform model with the unigram model and reevaluate it using the evaluation texts.

The bigram model is then added to the mix. Similarly, each model in this three-model interpolation will have the same interpolation weight of 1/3. We continue to add greater *n*-gram models to the mix while maintaining the same mixture weights across models.

Step 1: set the weight of each *n*-gram model to a number between 0 and 1, so that the total is less than 1.
Step 2: the goal function is differentiated with regard to each *n*-gram model weight (a1 to a5). The gradient of the objective function defined with respect to that of weight is often referred to as this derivative.
Step 3: each model's weight should be increased by a fraction of its gradient from Step 2. Because it influences how quickly the model weights are updated in each step, this fraction is frequently referred to as learning rate.
  (1) $$\begin{array}{c} a_{j}=a_{j}+\lambda \frac{\partial J}{\partial a_{j}}, \end{array}$$
where *j* = mapping cost, starts from 0 and increases during each iteration until average log likelihood reaches the max value.
Step 4: by subtracting the new *n*-gram model weights from 1, the uniform model's weight can be adjusted.
Step 5: finally, we repeat steps 2 and 3 until our average log likelihood has reached its maximum value.

RETRACTED

### 4.2. Training the Model

For a given *n*-gram model, we have the following.

1. The probability of each word is decided by the *n* − 1 words that are before it. In a trigram model (*n* = 3), for example, the probability of each word is determined by the two words that come before it.
2. The fraction of times this *n*-gram appears among all the preceding (*n* − 1)-grams in the training set is used to calculate this probability. To put it another way, training the *n*-gram model simply entails calculating these conditional probabilities based on the training text.

As a result, we can utilize the average log likelihood as the *n*-gram model's assessment metric once more. The stronger our *n*-gram model is, the higher the average probability it assigns to each word in the evaluation text.

More sophisticated methods for predicting the likelihood of a word *w* given a history *h*, or the probability of an entire word sequence *W*, will be required. To determine the probabilities of complete sequences such as *P* (*w*_1_, *w*_2_,…, *w*_*n*_), we must use the chain rule of probability to decompose the probability:

(2) $$\begin{array}{c} w_{ij}\left(t+1\right)=w_{ij}+\eta \frac{\partial \;\log\left(p\left(v\right)\right)}{\partial w_{ij}}. \end{array}$$

Now, by applying the chain rule to words, we get

(3) $$\begin{array}{c} P\left(w_{1:n}\right)=P\left(w_{1}\right)P\left(w_{3}|w_{1:2}\right)\ldots P\left(w_{n}|w_{1:n-1}\right)\\ =\prod_{k=1}^{n}P\left(w_{k}|w_{1:k-1}\right). \end{array}$$

The chain rule demonstrates the connection between computing a sequence's joint probability and computing a word's conditional probability given prior words. (3) implies that by multiplying a number of conditional probabilities together, we may estimate the joint probability of an entire sequence of words.

The proposed *n*-gram model is based on the idea that rather than assessing a word's likelihood based on its whole history, we can approximate it using only the latest few words. The bigram model uses only the conditional probability of the preceding word *P* (*w*_*n*_|*w*_*n*−1_) to approximate the probability of a word given all previous words *P* (*w*_*n*_|*w*_1_:*n* − 1). A Markov assumption states that the probability of a word is exclusively controlled by the preceding word. Markov models are a type of probabilistic model that assumes we can anticipate the likelihood of a future unit without having to look too far back in time. As a result, the general equation for this *n*-gram approximation of the conditional probability of the following word in a sequence is

(4) $$\begin{array}{c} P\left(w_{n}|w_{1:n-1}\right)\approx P\left(w_{n}|w_{n-N+1:n-1}\right). \end{array}$$

Maximum likelihood estimation, or MLE, is a simple method for estimating probabilities. By taking counts from a corpus and normalizing them to fall between 0 and 1, we can get the MLE estimate for the parameters of an *n*-gram model. The program can extract *n*-grams at both the character and word level. Other settings in this method can be predetermined, such as omitting stop words and non-ASCII letters as well.

RETRACTED

Tokenizing strings is the process of converting strings into tokens. Separate strings are detected and labelled with a unique ID in this way. Token separators are frequently perceived as white spaces and punctuation marks. Tokens that appear frequently in the data are given a lower weight than tokens that appear infrequently. Each token represents a feature, which is represented by a feature vector. A multivariate sample is a vector that comprises all of the features for a specific document. Thus, vectorization is the generic process of converting textual data into numerical feature vectors that machine learning algorithms can handle. Setting the rules and training the neural network for classifying streaming data forms the second phase of the work and is discussed in detail in the next section.

The primary principle behind utilizing *N*-grams to generate text is to presume that the last word (*x*_*n*_) of an *n*-gram may be deduced from the previous words in the same *n*-gram (*x*_*n*−1_, *x*_*n*−2_,…, *x*_1_), which is known as context. So the model's basic premise is that in order to forecast the next word, we do not need to maintain track of the entire phrase; instead, we just need to look back for *n* − 1 tokens.

## 5. Deep Belief Neural Network for Classification

A deep belief neural network (DBN) may learn to probabilistically recreate its inputs when trained on a set of examples without supervision. After that, the layers serve as feature detectors. A DBN can be further taught under supervision to do categorization after completing this learning stage [27]. DBNs are made up of simple, unsupervised networks like restricted Boltzmann machines (RBMs) or autoencoders, with the hidden layer of each subnetwork serving as the visible layer for the next. A generative energy-based undirected model with a “visible” input layer and a “hidden” layer, as well as connections between but not within layers, is known as an RBM. This results in a quick, unsupervised layer-by-layer training approach, in which contrastive divergence is applied to each subnetwork in turn, starting with the “lowest” pair of layers as shown in Figure 4.

RETRACTED

The contrastive divergence approach is used to speed up the learning for an RBM, and the fundamental idea is to update all of the hidden units in parallel, starting with visible units, reconstructing visible units from the hidden units, and then updating the hidden units again. Layers of stochastic binary units with weighted connections make up a basic belief network. Furthermore, because the network is an acyclic graph, we can see what kinds of data the belief network believes in at the leaf nodes. The goal of a belief network is to infer the states of unseen stochastic binary units and adjust the weights between them so that the network can provide data that are equivalent to what is observed. The stochastic binary units in belief networks have a state of 0 or 1, with the probability of reaching 1 controlled by a bias and weighted input from other units. This is represented as

(5) $$\begin{array}{c} w_{ij}\left(t+1\right)=w_{ij}+\eta \frac{\partial \;\log\left(p\left(v\right)\right)}{\partial w_{ij}}. \end{array}$$

Here *p* (*v*) corresponds to the probability of a visible vector, *ƞ* represents the learning rate, and *W* is the weight matrix between the hidden (*i*) and visible layers (*j*). The contrastive divergence (CD) technique is used to learn a layer of features from visible units as the initial stage in training DBN [28]. The next stage is to treat previously learnt features' activations as visible units and learn features from a second hidden layer. When the learning for the final hidden layer is completed, the entire DBN is trained. DBN may be trained using this simple greedy learning technique. This is because the CD algorithm in the training RBM seeks for the local optimum for each layer, and the following stacked RBM layer takes those optimally trained values and looks for the local optimum again. As each layer is continually educated to achieve the best value, the global optimum is likely to emerge at the end of this method.

We can employ persistent contrastive divergence because the sampling caused by contrastive divergence greatly biases the samples from the model distribution toward the most recent data. New samples are produced at each iteration by sampling conditioned on the most recently sampled hidden states, which are retained between data points, and the model distribution is randomly initialized.

RETRACTED

By stacking RBMs and interpreting the hidden layer of the lower RBM as the visible layer of the next layer, DBNs can be created. It has been demonstrated that adding hidden layers and using the previously stated unsupervised learning methods for RBMs will enhance the lower bound on the training data's log-likelihood. Higher layers are more likely to encode abstract features, which are usually extremely useful for classification applications. After that, supervised learning methods can be used to train the DBN's top layer, and error backpropagation can be used to optimize the entire multilayer network for the job. DBNs can also be used to link together distinct sets of data. Preprocessing hierarchies for both inputs may be created independently in this case, and the top levels of both hierarchies can be considered as a shared visible layer for a new association layer to be formed on top of them. As a result, DBNs can have tree-like structures as well as single hierarchies.

Data labelling by hand is both costly and time-consuming. We can use pseudo labelling to label our data to speed up the process of labelling it as shown in Figure 5. Pseudo labelling is a semisupervised labelling technique that still requires labelled data. Machine learning methods are used to develop models in pseudo labelling. As a class of unlabeled data, the model was then utilized to construct a pseudo label.

We utilized multinomial Nave Bayes as a model in this study. In this work, we created our sentiment analysis model by performing several experimental model variations. We built the first model variations using deep belief neural network. We also compared the accuracy of the three algorithms by using term frequency-inversed document frequency (TF-IDF) as a characteristic instead of TFIDF. Several deep neural network methods, including convolutional neural network (CNN) and long short-term memory (LSTM), were used to create the second sentiment analysis model variations (LSTM).

The major purpose of this project's exploratory data analysis phase was to become familiar with the data frame's columns and begin developing research ideas. Starting with the phase of importing the data with pandas, we can see that all of the following information is available for each tweet and that includes user name, description, followers, friends, favourites, id, date, text, hashtags, sources, and retweets. The depth of a convolution neural network suffers from overfitting due to the necessity to train a large number of hyper parameters. Dropout regularization is applied to completely linked layers to solve the problem of a large number of concealed units and their connections. Two key metrics, namely the polarity and subjectivity, are calculated. By sorting the data set by polarity scores and then presenting the top rows, we may examine these types of tweets and complete the sentimental analysis.

RETRACTED

## 6. Results and Discussion

The easiest approach to assess a language model's performance is to embed it in an application and track how much the application improves. Extrinsic evaluation refers to this type of end-to-end assessment. Extrinsic evaluation is the only way to determine whether a certain component change will actually help with the task at hand. An intrinsic evaluation metric is one that assesses a model's quality without regard to its application. A test set is required for an intrinsic evaluation of a language model. The probabilities of an *n*-gram model, like many other statistical models in our field, are derived from the training set or training corpus on which it is trained. The performance of an *n*-gram model on unseen data, referred to as the test set or test corpus, can subsequently be used to assess its quality.

The research focuses on sentiment analysis of Twitter messages utilizing the Python programming language with the Tweepy and TextBlob libraries. Tweepy allows us to find relevant information by using keywords, hashtags, timelines, trends, or geolocation. For searching the tweets with the COVID hashtag, the following command is used.

  api = tweepy.API(auth, wait_on_rate_limit = True) #important.
  self.tweets = tweepy.Cursor(api.search, *q* = 'COVID-19, lang = ”en”).items(100)

The prepared dataset, which included positive, negative, and neutral classes, was used in the experiments. A total of 47,000 tweets were used in the training process, with 11,000 being used in the testing cycle. Different *N*-gram models were combined with a set of classifiers in the suggested strategy in Table 1.

In order to determine the best settings for the preprocessing approaches and classifiers, we ran a series of experiments to see which alternatives would yield the most accurate results.  Section 3 includes a detailed description of the chosen preprocessing methods. Some of the sample tweets are listed below in Table 2 with corresponding sentiment category.

We notice that when we select qualities with an information benefit greater than zero, the number of them is reduced significantly. We chose around 70% of the attributes ranked as more deserving for the second feature extraction, where the attributes are analysed using the random forest algorithm. The suggested classifier accuracy is compared to other techniques in the literature in Table 3.

Table 3 shows how classifier performance varies based on the preprocessing methods used. The behaviour of dataset representations is not consistent. There is no representation that consistently produces better results when compared to others. In general, 1-to-3-grams outperform the other formats; however, they are a close second to unigram.

RETRACTED

The attribute selection process enhances classification performance when compared to picking all attributes, according to our findings. This results from the elimination of redundant and irrelevant features from datasets, which can lead to overfitting by deceptive modelling techniques.  Table 4 shows the general community sentiment for the study period, organized by sentiment words. It demonstrates that in March and April, the public had a very favourable attitude. Late May saw a minor decrease, followed by a substantial decrease in June. This could be attributable to an increase in COVID-19 confirmed cases. There were peaks and valleys in negative sentiment.

Some words, such as “coronavirus” and “Wuhan,” have the highest frequency in our database. In the tweets column, there are a variety of #hashtags. However, they are nearly same in all attitudes; therefore, they are unable to provide us with useful information. The efficiency of the proposed algorithm is shown in Figure 6 when compared to other categorization methods in the literature.

It is evident from Figure 6 that the proposed method outweighs the other existing methods in the literature in terms of classifier accuracy. The number of repetitions also affects classification accuracy. As the number of iterations is impacted by the size of the experiment, we chose iteration = 50, 100, 150, 200, and 300 and then manually examined the data throughout each iteration. The results reveal that in the range from 100 to 200 iterations, there is no significant change. As a result, we limited our model to 150 iterations. While sentiment analysis of tweets can reflect public opinion, it cannot express the true impact of the virus, as evidenced by the rapidly increasing number of cases and deaths every day.

## 7. Conclusion

With the rise in popularity of social networking sites, they have become a strong tool for influencing people and disseminating information to the general public. However, due to the lack of contextual information in the texts, sentiment analysis for brief texts such as Twitter is particularly difficult. As a result, numerous algorithms are always being created in order to achieve the finest sentiment analysis model result. A preliminary phase of text preprocessing and feature extraction is required to complete the classification operation. Because preprocessing activities have an impact on classification quality, we run a number of experiments on various generated datasets. Deep belief networks are a type of deep architectural network that is constructed from stacks of restricted Boltzmann machines. DBNs may also be utilized for tasks in both an unsupervised and supervised situation, and they take full advantage of outstanding techniques like unsupervised pretraining and fine tuning on a downstream job. The results of our research show that by selecting and representing features correctly, sentiment analysis accuracy can be increased. The produced datasets were analysed in terms of positive and negative attitudes, fear, and trust emotions expressed in the tweets. To avert anarchy and panic, policymakers can adopt public opinion surveillance techniques. For well-intentioned data, Twitter can be used. All governments can benefit from timely awareness of public mood in order to establish an effective strategy for better managing the situation and a communication strategy for disseminating accurate and trustworthy information and engaging the public in the appropriate response activities. This will be our future directions as well. In future, additional twitter data can be considered for experimentation. The impact of COVID-19 on financial sector, employability, and personal life of the individuals may be analysed and prediction will be performed using machine learning techniques.

RETRACTED

## Figures and Tables

**Figure 1:** A typical framework with supervised learning model for text classification.

**Figure 2:** Sentimental analysis pipeline.

**Figure 3:** *N*-grams model for generative applications.

**Figure 4:** DBN learning architecture with two hidden layers and one output layer.

**Figure 5:** Labelling method.

**Figure 6:** Classifier accuracy between proposed and literature methods.

**Table 1:** Statistics overview of the tweets COVID-19 dataset.

Feature	Total	Unique	Percentage of tweets (%)
Hashtag	3653928	566308	30
Mention	5363449	1251963	40
Entity	11537537	331307	70

**Table 2:** Sample tweets classification from the data set.

Sample tweet	Sentiment category
Bright vision, a community hospital, is transferring all patients to create room for stable COVID-19 cases.	Mixed sentiment
Any fellow patriot who celebrates Boris contracting the Corona virus is a complete cunt.	Negative/sad
Twittizens, good morning I wish you a day without coronas.	Positive/joy
Perhaps if I lock my front door, the coronavirus will be kept away.	Anger
In order to infect visitors with malware, hackers create false coronavirus maps.	Fear
My heart hurts so much at the notion of Jacob's Nashville performance being cancelled. Please go away.	Negative/sad

RETRACTED

**Table 3:** Classifier accuracy comparison with the proposed method.

*N*-gram	Type of attribute	Classifier accuracy			
		Proposed DBN (%)	Naïve Bayes (%)	SVM (%)	K-nearest neighbors (%)
Unigram	All twitter data	80.3	79.4	81.9	73.3
	Information gain >0	84.1	86.6	83.6	74.2
	Best 70% on ranking	88.1	88.0	83.2	73.5

Bigram	All twitter data	86.1	75.2	85.8	62.7
	Information gain >0	90.3	89.0	82.8	63.3
	Best 70% on ranking	89.5	83.0	87.8	62.7

1 to 3 gram	All twitter data	86.1	85.7	82.5	68.8
	Information gain >0	90.1	92.5	84.1	66.0
	Best 70% on ranking	89.0	88.3	83.8	66.4

**Table 4:** Words classification based on different sentiments across time periods.

Sentiment	March 2020	April 2020	May 2020	June 2020
Positive	32430	32437	31572	26507
Negative	34181	31538	37410	20677
Fear	31496	35542	34982	29184
Noncategorized	136916	155750	147115	101254
Total	235023	255267	251079	177622

## Data Availability

The data used to support the findings of this study are available from the corresponding author upon request.
